# An Improved Double Channel Long Short-Term Memory Model for Medical Text Classification

**DOI:** 10.1155/2021/6664893

**Published:** 2021-02-23

**Authors:** Shengbin Liang, Xinan Chen, Jixin Ma, Wencai Du, Huawei Ma

**Affiliations:** ^1^School of Software, Henan University, Kaifeng, China; ^2^Institute of Data Science, City University of Macau, Taipa, Macau, China; ^3^School of Computing and Mathematical Science, The University of Greenwich, London, UK; ^4^School of Information Technology, Beijing Institute of Technology, Zhuhai, China

## Abstract

There are a large number of symptom consultation texts in medical and healthcare Internet communities, and Chinese health segmentation is more complex, which leads to the low accuracy of the existing algorithms for medical text classification. The deep learning model has advantages in extracting abstract features of text effectively. However, for a large number of samples of complex text data, especially for words with ambiguous meanings in the field of Chinese medical diagnosis, the word-level neural network model is insufficient. Therefore, in order to solve the triage and precise treatment of patients, we present an improved Double Channel (DC) mechanism as a significant enhancement to Long Short-Term Memory (LSTM). In this DC mechanism, two channels are used to receive word-level and char-level embedding, respectively, at the same time. Hybrid attention is proposed to combine the current time output with the current time unit state and then using attention to calculate the weight. By calculating the probability distribution of each timestep input data weight, the weight score is obtained, and then weighted summation is performed. At last, the data input by each timestep is subjected to trade-off learning to improve the generalization ability of the model learning. Moreover, we conduct an extensive performance evaluation on two different datasets: cMedQA and Sentiment140. The experimental results show that the DC-LSTM model proposed in this paper has significantly superior accuracy and ROC compared with the basic CNN-LSTM model.

## 1. Introduction

People consult medical experts online in healthcare communities and ask for treatment plans through symptom description or seek the recommended hospital and department. Using a deep learning algorithm to classify disease symptom text can optimize the allocation of medical resources and improve the efficiency of medical treatment. Text categorization is a classic problem in the field of Natural Language Processing (NLP). For an effective medical diagnosis, we proposed the idea of using an improved LSTM model to implement medical consultation text classification. The commonly used classification methods include Naïve Bayes [1], Support Vector Machine (SVM) [2], and Decision Trees [3]. These classic machine learning classification algorithms have achieved significant results in text classification tasks. With the research and development of neural networks and deep learning, Convolutional Neural Network (CNN) and Recurrent Neural Network (RNN) have been found to exhibit excellent performance in text classification tasks. At the same time, some models of Chinese question and answer in the medical field have been proposed. Jain and Dodiya [4] have proposed a rule-based framework for the medical question-answering system. Yin et al. [5] designed an algorithm for clustering and similarity evaluation of similar questions and answers for the problem of low efficiency of online healthcare consultation. Feng et al. [6] used CNNs to learn the representation of question and answer combination and further used it to calculate different questions and candidates. Zhang et al. [7] proposed an end-to-end word embedding multiscale CNN model for question and answer matching in the medical field.

Our primary contribution is a new Double Channel LSTM model, called DC-LSTM, and we add a hybrid attention mechanism to LSTM, which can selectively learn long sequences and make deep neural networks in each batch of training. This proposed model can learn different forms of features, enhance model learning and expression skills, and prevent overfitting. The experimental results show that the DC-LSTM model can significantly improve the accuracy compared with other CNN or RNN models. Particularly in the medical diagnosis classification, using this model can help people quickly choose the right outpatient department for medical treatment and improve the efficiency of outpatient service.

## 2. Related Work

CNN and RNN are two typical deep neural network models. CNN is typically applied in image processing [8] and speech recognition [9], while RNN is usually applied in machine translation and text sequence problem [10]. At the same time, some improved models have been derived. The LSTM proposed by Hochreiter and Schmidhuber in 1997 [11], which is based on the RNN-derived network model, is suitable for processing and predicting important tasks with relatively long intervals and delays in time series.

### 2.1. CNN Model

CNN is a common deep learning network architecture. Hubel and Wiesel are inspired by the natural visual cognitive mechanism of biology. With the improvement of data volume and computing power, CNN has become a research hotspot in recent years. CNN consists of convolution, activation, and pooling layer. Many researchers have proposed some improved CNN models in text classification, such as fastText [12], textCNN [13], and Bi-LSTM [14,15], which are very effective, but they still have some problems such as generality and difficulty in extracting specific context features.

### 2.2. Convolutional Layer

Convolution is the most basic operation in CNN, each convolutional layer is composed of several convolution units, and the parameters of each convolution unit are optimized by a backpropagation algorithm. The purpose of convolution operation is to extract different features of input. More layers of network can extract more complex features from low-level features iteratively. The convolution kernel can scan the input features according to a certain law and multiply the input features by matrix elements in the receptive field and then sum all the results and add the bias. The formula used is as shown in

(1) $$\begin{array}{c} Z^{l+1}\left(i,j\right)=\left[Z^{l}⊗w^{l}\right]\left(i,j\right)+b=\sum_{k=1}^{K_{l}}\sum_{x=1}^{f}\sum_{y=1}^{f}Z_{k}^{l}\left[\left(s_{0}i+x,s_{0}j+y\right)w_{k}^{l+1}\left(x,y\right)\right]+b,\;\left(i,j\right)\in \left\{0,1,\ldots ,L_{l+1}\right\},\\ L_{l+1}=\frac{L_{l}+2p-f}{s_{0}}+1, \end{array}$$

where *b* is the amount of deviation; *z*^*l*^ and *z*^*l+*1^ represent the input and output of the *l* *+* 1th convolution layer; *L*^*l*+1^ is the size of *Z*^*l*+1^; *Z* (*i*, *j*) is the corresponding feature matrix; *f* is the size of convolution Kernel; *s*_0_ is the step size of convolution; and *p* is the padding number.

### 2.3. Pooling Layer

After the feature extraction of the convolutional layer, the output feature matrix is passed to the pooling layer for further feature extraction and information filtering. The pooling layer contains a preset pooling function, which can use the features of its neighboring regions in the feature matrix. The statistics are replaced, and the definition of pooling is as shown in

(2) $$\begin{array}{c} A_{k}^{l}\left(i,j\right)={\left[\sum_{x=1}^{f}\sum_{y=1}^{f}A_{k}^{l}{\left(s_{0}i+x,s_{0}j+y\right)}^{p}\right]}^{1/p}, \end{array}$$

where *s*_0_ is the size of the pooling step and *p* is the parameter that has been customized specifically. When *p* = 1, this is called average pooling, and when *k* ⟶ ∞, this is called maximum pooling.

### 2.4. LSTM Model

LSTM is a special RNN structure that can learn long-term dependencies. RNN can propagate historical information through chained neural network architecture. When processing sequential data, it looks at the current input *x*_*t*_ and the previous output of the hidden state *h*_*t*−1_ for each time step. However, as the gap between the two-time steps becomes larger, the traditional RNN that can learn the long-term dependency characteristics becomes more difficult. The LSTM proposal addresses this long-term dependency problem and has achieved significant good performance in the statistical machine translation task of Chen et al. [15], making LSTM a successful model. The structure of the LSTM model is shown in Figure 1.

The LSTM architecture provides a series of repeating modules for each time step in a standard RNN. These modules are called cells. At each time step, the output of the module is controlled by a set of gates in *R*_*d*_ as a function of the old hidden state *h*_*t*−1_ and an input of the current time step *x*_*t*_ described as follows: forget the gate *f*_*t*_, input the gate *i*_*t*_, and output the gate *o*_*t*_. These gates together determine how to update the current memory unit *c*_*t*_ and the current hidden state *h*_*t*_. We use *d* to represent the memory dimension in LSTM, and all vectors in this architecture share the same dimension. The LSTM conversion functions are defined as follows:

(3) $$\begin{array}{c} i_{t}=\sigma \left(W_{i}\cdot \left[h_{t-1},x_{t}\right]+b_{i}\right),\\ f_{t}=\sigma \left(W_{f}\cdot \left[h_{t-1},x_{t}\right]+b_{f}\right),\\ q_{t}=\tanh\left(W_{q}\cdot \left[h_{t-1},x_{t}\right]+b_{q}\right),\\ o_{t}=\sigma \left(W_{o}\cdot \left[h_{t-1},x_{t}\right]+b_{o}\right),\\ c_{t}=f_{t}\cdot c_{t-1}+i_{t}\cdot q_{t},\\ h_{t}=o_{t}\cdot \;\tanh\left(c_{t}\right), \end{array}$$

where *σ* is a logical sigmoid function whose output is [0, 1], tanh represents a hyperbolic tangent function, and its output is [−1, 1]. LSTM is specifically designed to learn time-series data for long-term dependencies, so we chose LSTM on the convolutional layer to learn this dependency in higher-level feature sequences.

### 2.5. Word Embedding

Glove is also known as Global Vectors for word representation [16]. It is a word representation tool that is count-based and uses overall statistics. A vector of real numbers is obtained that captures some semantic properties between words, such as similarity and analogy. We can calculate the semantic similarity between two words by computing the vector, such as Euclidean distance or cosine similarity.

Word2Vec is a three-layer neural network, which consists of the input layer, the hidden layer, and the softmax layer. The training process is to train the central words and context words by constructing a fake supervised task called Fake Task. The middle-hidden layer weight is used as a trained word vector. According to the size of the input and output data, it has two methods: Skip-Gram method and CBOW method. The former method uses the central word as input and uses the context word of the central word as the label to be predicted for training. The latter method is just the opposite, using the context word as input. As the input data, the context word is trained with the central word as the output to be predicted. After the training is completed, the output information is discarded, and the weight of the middle layer is used as the trained word vector. The Word2Vec model solves the computational bottleneck in the NNLM model. It can easily process tens of millions of text data and can use variable-length sequences as input. With this advantage, the neural network model can model more complex contexts, and Word vectors can contain richer semantic information.

## 3. Methodology

Traditional CNN and RNN networks often only use word-level embedding, and the semantic features are limited. These traditional models have a very limited capability, especially for words that need to use context to determine semantics. Therefore, it is necessary to expand channels and use multilevel embedding to improve input characteristic diversity. At the same time, the relative importance of each word in the text is different for the modality expressed. Some words contribute more to the modality, some words have less contribution to the modality, and the emotions expressed by each word are also prioritized. Therefore, in order to solve the problem of not being able to selectively learn the emotional characteristics of each word, we can add hybrid attention after LSTM and make trade-offs for different words with different emotions, improve the learning ability of LSTM model, and improve the special characteristics of neural network learning. This creates the ability to simultaneously improve generalization and prevent overfitting from occurring. The model is divided into three parts of CNN-LSTM, Double Channel, and hybrid attention, of which Double Channel is the most important structure.

### 3.1. CNN-LSTM

In our work, we use both CNN and LSTM. The improved CNN structure in our model is similar to ConvNets proposed by Zhang et al. [17] in 2015. The ConvNets consists of nine layers deep with six convolutional layers and three fully connected layers. The structure of the ConvNets is shown in Figure 2.

On the other hand, RNNs have been widely exploited to deal with variable-length sequence input. However, when the length of the input sequence becomes longer, CNNs may suffer from a gradient problem of disappearing or exploding, which will make it more difficult to learn information from a longer time context. LSTM is one of the popular variations of RNN which is proposed to solve this problem. Its network solves this problem by introducing a gate structure in each LSTM unit. The forgetting gate decides what information to be discarded from a cell state and how many new inputs are determined by the input gate. The information is added to the cell state, and the output gate determines what value to be output based on the current state of the cell.

We introduce the Double Channel mechanism in the CNN-LSTM model and input multiple levels of embeddings at the same time to acquire multiple levels of features, in order to solve the problem that the word-level and character-level features cannot be extracted at the same time.

In this model, according to the embedding granularity that is used, the structure is divided into Char-Channel and Word-Channel. The model structure is the same in each channel, which is divided into two parts: CNN and LSTM neural network. In the CNN part, the convolution result *c* is calculated for the input sequence *X* and the convolution kernel *K*,

(4) $$\begin{array}{c} c=\text{conv}\left(X,K\right)+b. \end{array}$$

For the above LSTM calculation process, in order to simplify the formulation, it is unified as LSTM (x). For the convolution neural network and long-term and short-term memory neural network, there are two kinds of structures that can be used: series and parallel. At present, the most commonly used structure is series structure, but there is the information loss phenomenon with this, because information compression and loss will occur in the convolution process. The long-term and short-term memory neural network also receives compressed information and loses most of the time-series characteristics with the series structure. It is unable to give full play to the advantages of LSTM. To solve this problem, the parallel structure is chosen over the series structure and the results are mosaic. At the same time, the structure in each channel is recorded as

(5) $$\begin{array}{c} \text{channel}\left(x\right)=\left[\text{conv}\left(x\right)\;⊕\text{ LSTM}\left(x\right)\right]. \end{array}$$

From equation (5), we can get the basic description of Char-Channel and Word-Channel. Their input is corpus *x*, and the output is *C*_out_ and *W*_out_, respectively,

(6) $$\begin{array}{c} C_{\text{out}}={\text{channel}}_{\text{emb}=V_{e}}\left(x\right), \end{array}$$

(7) $$\begin{array}{c} W_{\text{out}}={\text{channel}}_{\text{emb}=V_{g}}\left(x\right). \end{array}$$

*V*_*e*_ and *V*_*g*_ in equations (6) and (7) are the word-level embedding vectors trained and the char-level embedding vector. We concatenate the results of the two channel outputs as a hidden layer output,

(8) $$\begin{array}{c} h=\left[c_{\text{out}}\;⊕\;w_{\text{out}}\right]. \end{array}$$

Then, the result of the hidden layer is sent to the fully connected layer, and then the softmax layer is used for classification output,

(9) $$\begin{array}{c} \hat{y}=\text{softmax}\left(\text{dense}\left(h\right)\right). \end{array}$$

The Double Channel structure is as shown in Figure 3.

### 3.2. Hybrid Attention

The weight score *ω* is an important component of the dynamic adaptive weight, and its calculation method is as shown in equations (10) and (11):

(10) $$\begin{array}{c} e_{i}=v_{a}^{T}\tanh\left(W_{a}h_{i}+b\right), \end{array}$$

(11) $$\begin{array}{c} h_{i}=\langle h_{t}^{\prime }\;:c_{t}\rangle , \end{array}$$

where *h*_*t*_′ is the LSTM output at time *t*, *c*_*t*_ is the status in LSTM at time *t*, *h* is the hidden layer output, *w*_*a*_ is the random initialization weight matrix, *v*_*a*_ is the random initialization vector, and *b* is the random initialized bias. Next, the score *ω* is calculated as shown in

(12) $$\begin{array}{c} \omega =\frac{\exp\left(e_{i}\right)}{\sum_{k=1}^{T_{x}}\exp\left(e_{i}k\right)}, \end{array}$$

where *x* is the length of the sequence.

The output vector *c*_*i*_ weighted by the dynamic adaptive weight, as shown in

(13) $$\begin{array}{c} c_{i}=\sum_{j=1}^{T_{x}}\omega \cdot h_{j}. \end{array}$$

### 3.3. DC-LSTM Overview

In order to better obtain semantic representation and extract text features, we have designed DC-LSTM using the convolution layer through first embedding the input text sequence, then obtaining the vector representation of these sequences, and finally convolving the sequence using the convolution layer. This model can extract word-level semantic features and the pool, reduce the input data and the output size, and also reduce the risk of overfitting. The data processed by the convolution layer is sent to the LSTM layer, and the LSTM can analyze the timing characteristics in the data. This algorithm can extract some information of context semantics, ignore secondary information, and ensure the accuracy of classification tasks. The DC-LSTM model is shown in Figure 4.

## 4. Experiments

In order to verify the reliability of the model, a complete contrast experiment was designed. The two datasets of cMedQA and Sentiment140 were used to compare the DC-LSTM model and the basic CNN-LSTM model proposed in this paper was used.

### 4.1. Datasets

To better validate the model's effects, the cMedQA medical diagnosis dataset and the Sentiment140 Twitter dataset are used for verification experiments. The cMedQA dataset is a Chinese text dataset with 792,099 medical consultations which include Andriatria, Internal Medicine, OAGD, Oncology, Pediatric, and Surgical department. The distribution of cMedQA is shown in Figure 5. The question-answering pairs have been preprocessed and classified into different categories. Each pair of QA is encoded as a series.

Meanwhile, to verify the model's good generality, we also select another dataset unrelated to medicine: Sentiment140. Sentiment140 dataset is a tweeter sentiment analysis dataset created and organized by three computer science students from Stanford University, Alec Go, Richa Bhayani, and Lei Huang, with 1.6 million training data and 498 test data. These data are divided into negative, neutral, and positive categories according to emotional polarity. The detailed description of these two datasets is shown in Table 1.

Some samples in cMedQA dataset are as shown in Table 2.

As we can see from Table 2, the dataset includes three main features, namely, department, title, and ask. Title and ask indicate the consultant's symptoms, while department is the answer which indicates the department of treatment. Title points out the core demands of consultants, while ask further describes the content of demands, which puts forward higher requirements for the ability of the model to explain the context.

### 4.2. Evaluation

The evaluation indicators use the accuracy rate, precision rate, recall rate, and F_1_-score to measure the performance of the model.

Define TP is True Positive, FP is False Positive, TN is True Negative, FN is False Negative, and then

(14) $$\begin{array}{c} \text{precision}=\frac{\text{TP}}{\text{TP}+\text{FP}},\\ \text{recall}=\frac{\text{TP}}{\text{TP}+\text{FN}}\text{,}\\ \text{accuracy}=\frac{\text{TP}+\text{TN}}{\text{TP}+\text{FP}+\text{TN}+\text{FN}}\text{.} \end{array}$$

Accuracy refers to the proportion of correctly predicted samples to all samples, precision refers to the proportion of samples that are positively positive, recall refers to the proportion of all positive samples that are correctly predicted, and F_1_-score refers to the harmonic average of precision and recall.

### 4.3. Hyperparameter

It is well known that the quality of hyperparameters will directly affect the training effect of the model, so it is important to choose a series of optimal hyperparameters. The settings of the hyperparameters are shown in Table 3.

### 4.4. Experiment Results

This section compares experiments and uses our proposed improved model, DC-LSTM, to compare it with CNN, LSTM, CNN-LSTM, and GRU models. The environment used in this paper is based on Tensorflow [18] as the background of Keras as the development verification environment, CUDA [19] as the GPU acceleration environment, and cuDNN [20] as the numerical computing environment of the deep neural network. The experimental results are shown in Table 4.

It can be seen from Table 4 that the DC-LSTM model proposed in this paper is superior to other models such as CNN, LSTM, CNN-LSTM, and GRU in terms of accuracy, precision, recall, and *F*_1_-score on cMedQA dataset and Sentiment140 dataset. The model has good generalization ability, and the model not only performs well in medical field but also performs better in other datasets.  Figure 6 further shows that the AUC value of DC-LSTM model on various outpatient data of cMedQA is higher than 0.9, which is also significantly higher than other models. In general, the improved model DC-LSTM has been improved in many evaluation indexes. This is due to the introduction of a multichannel mechanism, which can make full use of the attention mechanism's ability to calculate text weight and also make use of the powerful temporal feature learning ability of LSTM. In the channel, learning the semantic information carried by word vector and character vector can learn more features and more fine-grained features.

## 5. Conclusions

In this paper, we find that the basic CNN-LSTM model cannot perform differential learning when dealing with complex long-sequence data. After analyzing the possible causes, we propose an improved method, called DC-LSTM, which incorporates multiplication by weights (*w*) according to each time step of the sequence. The upper bias calculates the weight score, calculates the probability distribution of the weight score, and adds the hybrid attention according to the probability distribution. Experiments results have shown that DC-LSTM can effectively distinguish the emotional level of different words in sentences and assign different learning weights to different words, so that it can learn the sentiment features of each word in a differentiated way.

## Figures and Tables

**Figure 1:** Structure of LSTM.

**Figure 2:** Structure of ConvNets model.

**Figure 3:** The DC-LSTM structure.

**Figure 4:** DC-LSTM model.

**Figure 5:** Data statistics of cMedQA.

**Figure 6:** AUC value comparison of different models in cMedQA outpatient data.

**Table 1:** Overview of datasets.

Datasets	Number of training sets	Number of test sets	Categories	Features
cMedQA	792099	2500	6	3
Sentiment140	1600000	498	3	6

**Table 2:** Some samples in cMedQA.

Department(Answer)	Title	Ask
心血管科 Cardiovascular Department	高血压患者能吃党参吗? Can hypertensive patients take *Codonopsis pilosa?*	我有高血压这两天女婿来的时候给我拿了些党参泡水喝, 您好高血压可以吃党参吗? Hello, I am a hypertensive patient; my son-in-law gave me some *Codonopsis pilosa* as a gift, can I make tea with *Codonopsis pilosa*?
消化科 Digestive System Department	哪家医院能治胃反流 Which hospital can treat gastric reflux?	烧心, 打隔, 咳嗽低烧, 以有4年多 Heartburn, interval, cough, and low fever, more than 4 years

**Table 3:** Hyperparameter.

Items	Values
Word vector	Baidu Baike word + char 300d
Batch size	256
Filter size	3/5/7
Feature map number	150
Activation function	ReLU
LSTM output	128
Full connection layer output	200
Learning rate	Adadelta
Dropout	0.25
Loss	Binary crossentropy
Optimizer	Adam

**Table 4:** The results of the experiment.

Model	Dataset	Accuracy	Precision	Recall	*F*_1_-score
CNN	cMedQA	0.9570	0.8739	0.8803	0.8760
	Sentiment140	0.8831	0.8189	0.8188	0.8188

LSTM	cMedQA	0.9605	0.8857	0.8851	0.8852
	Sentiment140	0.9083	0.8255	0.8267	0.8256

CNN-LSTM	cMedQA	0.9615	0.8892	0.8898	0.8877
	Sentiment140	0.9010	0.8272	0.8271	0.8271

GRU	cMedQA	0.9611	0.8896	0.8795	0.8816
	Sentiment140	0.9044	0.8533	0.8532	0.8532

DC-LSTM	cMedQA	0.9729	0.9184	0.9183	0.9192
	Sentiment140	0.9112	0.8703	0.8703	0.8703

## Data Availability

The cMedQA data used to support the findings of this study have been deposited in the GitHub repository (https://github.com/liangsbin/Chinese-medical-dialogue-data). The Sentiment140 data used to support the findings of this study have been deposited in the Kaggle website (https://www.kaggle.com/kazanova/sentiment140).
